# Behavior and exocrine glands in the myrmecophilous beetle *Lomechusoides strumosus* (Fabricius, 1775) (formerly called *Lomechusa strumosa*) (Coleoptera: Staphylinidae: Aleocharinae)

**DOI:** 10.1371/journal.pone.0200309

**Published:** 2018-07-25

**Authors:** Bert Hölldobler, Christina L. Kwapich, Kevin L. Haight

**Affiliations:** 1 Social Insect Research Group, School of Life Sciences, Arizona State University, Tempe, Arizona, United States of America; 2 Biozentrum, Zoology II, University of Würzburg, Bavaria, Germany; University of Vienna, AUSTRIA

## Abstract

To become integrated into an ant society, myrmecophilous parasites must overcome both the defenses and the communication system of their hosts. Some aleocharine staphylinid beetles employ chemical and tactile strategies to invade colonies, where they later consume ant brood and participate in parasitic trophallaxis with host ants. By producing compounds that both appease their hosts and stimulate adoption, the beetles are able to live in and deposit their own eggs in the well defended ant nest. In the current paper, previous findings on the myrmecophilous behavior and morphological features of the staphylinid beetle *Lomechusoides* (formerly *Lomechusa*) *strumosus* are reviewed and re-evaluated. Hitherto unpublished results concerning the beetles’ ability to participate in the social food flow of their host ants are reported. Furthermore, we present an analysis and documentation of the behavioral interactions between beetles and host ants during the adoption process, and we report new histological and scanning electron microscopic analyses of the exocrine glands and morphological adaptations that underlie the myrmecophilous behavior of *L*. *strumosus*. The main features of *L*. *strumosus* are compared with those of the staphilinid myrmecophile *Lomechusa* (formerly *Atemeles*) *pubicollis*. The paper concludes with a description of the life trajectory of *L*. *strumosus* and presents a brief history and discussion of the hypotheses concerning the evolution of myrmecophily in *L*. *strumosus* and other highly adapted myrmecophilous parasites.

## Introduction

The ant colony and its immediate environment can be thought of as an ecological island, partitioned into many microhabitats that symbiotic organisms attempt to colonize [1–3]. Indeed, the ant colony and its surroundings are richly structured into many microhabitats such as foraging trunk routes, refuse areas, peripheral nest chambers, storage chambers, and brood chambers. These microhabitats are often occupied by a diversity of symbionts which exhibit special adaptations to each of the niches in turn [3–5]. Particularly, the brood chambers constitute an optimal niche within an ant nest for a social food-flow parasite, because there the food of highest quality is concentrated to be fed to the developing larvae, callow workers and queens. Moreover, the immature larvae in the brood chamber provide the most reliable prey for specialized myrmecophilous predators.

Nevertheless, in order to penetrate the brood chambers, which are defended by the ants, the myrmecophilous predator needs very special adaptations. This has been accomplished by some of the most evolutionarily advanced myrmecophilous staphylinids, of which the aleocharine beetle genera *Lomechusoides* and *Lomechusa* are premier examples [2, 6–11]. No one has published more papers or has observed *Lomechusoides strumosus* longer than Erich Wasmann has. Wasmann wrote more than 200 papers on myrmecophiles, most of them on *L*. *strumosus*. Much of this work is summarized in an overview published in 1915 [8]. In this paper, Wasmann critically responded to the publication of Karl Hermann Christian Jordan [6], who provided the first solid histological description of exocrine glands in adult *L*. *strumosus*. Jordan missed or misinterpreted several observations previously published by Wasmann, but was right to point out Wasmann’s histological misconceptions. Jordan was both the first to describe the peculiar defense gland in aleocharine beetles, and to recognize that the so-called trichomes in *Lomechusoides* and *Lomechusa* species are innervated and associated with exocrine glands (though his characterization of these glands was incorrect).

In the current paper, we re-visit *Lomechusoides strumosus* and re-examine the special exocrine glands and other morphological features that play a role in the beetle’s myrmecophilous behavior. We also investigate the behaviors associated with the process of beetle adoption, and the beetle’s participation in the social food flow of its host ants.

## Materials and methods

First a note concerning taxonomic confusion: In literally all behavioral studies and reviews dealing with mymecophiles of the genera *Lomechusoides* and *Lomechusa* from the past 100+ years (including the publications by Erich Wasmann, William Morton Wheeler, August Forel, Horace Donisthrope, Karl Escherich, Edward O. Wilson, David Kistner, Karl Hölldobler, Bert Hölldobler and many others) the genus *Lomechusoides* was called *Lomechusa*, and the genus *Lomechusa* was called *Atemeles*. A recent revision demonstrates that from a strict, taxonomic-priority point of view, this classification was wrong. To clarify the question of genus identity, we best cite a paragraph from the recent revision of the genus *Lomechusa* by Peter Hlaváč [12].

“The first species of the genus *Lomechusa* was described as *Staphylinus emarginatus* Paykull, 1789. Gravenhorst (1806) described the genus *Lomechusa* [with the type species *Lomechusa emarginata* (Payke) fixed by Latreille (1810)], and Dillwyn (1829) described the genus *Atemeles* [with the type species *Atemeles paradoxus* (Grav.)] subsequently designated by Westwood (1838). Later *Atemeles* was synonymized with *Lomechusa* (Blackwelder 1952: 226). Except for Brisout de Barneville (1860) all authors were using the generic name *Atemeles* for the species of *Lomechusa*, whereas the name *Lomechusa* was applied to species belonging to a different genus, which later was described as *Lomechusoides* by Tottenham (1939). Along with the description of a new genus (which included species related to *L*. *strumosus* Fabricius), Tottenham recognized the confusion around the generic names *Lomechusa* and *Atemeles* and clearly indicated that the names *Lomechusa* should be applied for all species related to *L*. *emarginata*. Unfortunately, subsequent authors (Palm 1949; Chilow 1977a, b, 1981 and Sawanda 1994) ignored this taxonomic act and the confusion has continued. Only recently new combinations for both genera have been done, for *Lomechusoides* (Maruyama & Hlaváč 2014) and also for *Lomechusa* (Smetana 2004).”

We fear that the confusion will continue, because, by far, more papers have been published concerning the behavioral interactions of these two aleocharine genera with their ant hosts applying the secondary, albeit taxonomically incorrect, nomenclature, than taxonomic studies of those genera, and even some contemporary taxonomic authors have used the old nomenclature [13–16] (cited in Hlaváč [12]. In this paper, we will use the generic names *Lomechusoides* and *Lomechusa* for what has been traditionally called *Lomechusa* and *Atemeles*, respectively.

Most of the data in this paper were collected in the years 1966, 1967, 1968 and 1969. *Lomechusoides* beetles were collected in the xerotherm limestone habitats of the lower Franconia surrounding of the river Main (Germany), from nests of the ant *Formica sanguinea*. In the laboratory, the beetles were housed in formicaria together with colonies of their host species, mainly *F*. *sanguinea*. The formicaria were constructed out of plaster of Paris casts, with various chambers. Typically, the ants housed their larvae in moist chambers and placed pupae in the dry chambers closer to the nest entrance. Each plaster nest was covered by a glass plate and located inside a Plexiglas box (26 X 20cm) (Fig 1), in which honey-sucrose water and chopped cockroaches (*Blatta germanica*) and mealworm larvae (*Tenebrio molitor*) as food were provided. We kept 12 such arrangements, but only 8 of the housed ant colonies had a queen.

**Fig 1:** Design of the laboratory formicarium for housing myrmecophile beetles and host ant colonies. The interconnected nest chambers are set in gypsum plaster and covered by a glass plate. The internal nest opens into an arena where food for the ants is provided and where beetles are placed for adoption experiments.

For adoption experiments, beetles collected in field colonies were placed in the arena close to the nest entrance and the behavioral interactions between ants and beetles observed. To obtain more quantitative behavioral data concerning the first interaction between beetle and host ants, we placed freshly collected beetles from field colonies into round, glass jars (9 cm in diameter, and 2.5 cm tall), with a moistened plaster floor, together with ten unfamiliar host-ant workers (n = 10 groups). Over a period of 15 minutes, we recorded the frequency of tactile interactions between ants and beetles. We noted the ants’ contact with the beetles’ abdominal posterior end, abdominal margin, head and legs, or any other body part.

Trophallaxis between the beetles and ants was measured by marking honey-sucrose-water (called in further mention “honey water”) with the radio isotope ^32^P, which was added as orthophosphate at a specific activity of 1–5 μc/mL. The liquid food was offered to the ants in small glass dishes. After feeding was completed, the ants were decontaminated by bathing them in distilled water. The ants were dried by placing them in a petri dish, the floor of which was covered with absorbent cellulose paper on which ants could walk around. After about 30 minutes, the ants were taken out. After each such maneuver, the petri dish was cleaned and new cellulose paper was put in. This procedure was first developed by Werner Kloft [17] and tested successfully in many subsequent tracer experiments with ants.

To measure the success of *Lomechusoides* beetles eliciting regurgitation from ant workers, two beetles were placed with 10 ants that had been fed ^32^P labeled honey-water in 10 x 10 x 5cm plastic boxes, the bottom of which was covered with fresh, slightly moistened filter paper. One day later, and at additional intervals, individual ants and beetles were measured separately. For measurements, we used a liquid scintillation counter with automatic sample changer (Philips, Eindhoven). However, we did not use liquid scintillation but instead placed individual live ants or beetles into the dry vials and measured the quantity of food by using the impulses per 100 seconds caused by Cherenkov radiation. In some cases, we also used an end-window counter. Bert Hölldobler was trained and certified to employ radioisotopes in biological studies at the University of Würzburg, Germany. He directed a licensed isotope laboratory at the Zoological Institute of the University in Frankfurt.

To test whether trophallaxis is offered based on the familiarity the ants have with particular *Lomechusoides* beetles, groups of 10 ants were given access to radioactively labeled honey water and placed with familiar or unfamiliar beetles. Nineteen such groups contained workers that were taken out of the nest in which the beetles had lived for at least one week, and 13 groups were composed of ants from foreign colonies (in part collected from nests in the field).

To determine whether beetles regurgitate food back to the ants or whether ants consume other secretions from the beetles, we placed beetles that had received radioactively labeled food from the host ants with unfed ants. In each trial, one beetle was placed with five ants 24-hr after feeding (n = 4 groups). The transfer of food from beetles to ants was monitored in 12-hr increments over 48 hours (n = 4 sampling events). The impulse counts for ants within each group were averaged during each sampling event. To determine whether beetles transferred food to ants over time, we used a linear mixed effects model that accounted for the repeated measuring of individuals during the four sampling bouts. The main and interactive effects of time and species identity (ant or beetle) on radioactive impulses/100 s represented fixed effects in our model, while group identity was a random effect (R v3.4.2, Packages: *Lme4*, *Lmertest*).

To test whether ants pick up feces or secretions from the abdominal tip of beetles, beetles were fed by ants with radioactively labeled honey-water. After 30–40 hours, the beetles were lightly touched with a soft water-color brush until they exuded a whitish secretion from the abdominal tip (n = 7). A pointed cotton bud was used to collect the secretion. Though, not our focus, beetles sometimes also discharged a strong-smelling secretion most likely from the defensive tergal gland during collection. We measured the radioactive imp/min for each cotton bud containing secretions, as well was an equal number of uncontaminated cotton buds, as a control. We used a paired t-test to determine if the secretion produced significantly more impulses/min than uncontaminated cotton buds. In these tests, we used an end window counter from Frieseke and Hoepfner (Erlangen).

For histological investigation, specimens were fixed in alcoholic Bouin (Dubosq Brasil) or Carnoy [18], embedded in methyl-methacrylate, and sectioned 5 μl thick with a Jung Tetrander microtome [19]. The staining was Hematoxylin-Eosin or Heidenhain Azan. All histological preparations, the radioactive tracer experiment, and the behavioral studies were conducted at the laboratory of B. Hölldobler at the University of Frankfurt. Re-analysis of the histological sections, SEM work, and the entire data analysis were carried out at the School of Life Sciences at Arizona State University.

## Results

### Exocrine glands

The subtribe Lomechusina of the tribe Lomechusini consists of three genera: *Lomechusa* (*Atemeles*), *Lomechusoides* (*Lomechusa*), and *Xenodusa*. A common feature of these three genera are the striking tufts of golden hairs on the lateral abdominal tergites II, III, IV, and V. These tufts are especially dense on the paratergites [6], (Fig 2). In contrast to Wasmann, Jordan recognized that these golden bristles are closely associated with exocrine glands, which open through the cuticle pores between adjacent golden bristles on the elevated edges of the paratergites and pleurites, and he recognized that the bristles are innervated. He described the glands as flask-shaped hypodermal gland cells. This characterization of the glandular cells cannot be confirmed by our investigations. Likewise, Pasteels [20], in his comparative study of exocrine glands of several aleocharine species, did not support these findings. Instead, our investigations clearly show that the “trichome cells” are secretory and the duct cells of which open in close vicinity of the trichome setae. Following the terminology of Noirot and Quennedey, and further specified by Billen [21, 22], these cells belong to class 3 (secretory cells associated with duct cells) (see also [11] for *Lomechusa*) (Figs 3 and 4). Such glandular cells also exist on the lateral regions of the tergites II, III, IV, and to a lesser degree in V (Fig 5). In addition, we found in each abdominal segment paired clusters of class 3 glandular cells, the ducts of which open through the cuticle of the lateral base of the tergal lobes near the spiracles. They are especially conspicuous in abdominal segments III, IV and V (Figs 3B and 4C). These glandular arrangements are identical in *Lomechusoides strumosus* and *Lomechusa pubicollis* and *L*. *emarginata*.

**Fig 2:** Scanning electron microscopic images of the abdomen of mymecophilous staphylinid beetles. Above: *Lomechusoides strumosus*; Below: *Lomechusa pubicollis*. AG indicates the lobes of the paratergites with the dense endowment with trichome hairs. This area is richly endowed with exocrine gland which are called “adoption glands”.

**Fig 3:** Adoption gland complex: Longitudinal section through the abdominal paratergal lobes of *Lomechusoides strumosus*. The picture above shows two lobes with trichome setae and glandular cells (GC). Below: The second major cluster of gland cells near the bases of the tergal lobes; the glandular ducts (GD) open through the cuticle near a tracheal tract. These glands are most likely part of the adoption gland complex.

**Fig 4:** Adoption gland complex: Longitudinal section through the abdominal paratergal lobes of *Lomechusa pubicollis*. (a) A lobe with trichomes and many glandular cells (GC), the ducts (GD) of which open through cuticle channels between the trichome setae. (b) Some areas of the lobes which have no trichomes, have glandular epithelia (GE) the cells of which open through cuticle channels (CuC). (c) The second cluster of gland cells on the bases of the trichome lobes the ducts of which open through the cuticle near a major tracheal tract.

**Fig 5:** Transversal section through the lateral edge of the abdominal tergites adjacent to a paratergal trichome lobe of *Lomechusoides strumosus*. Although in this part of the adoption gland complex trichome setae are sparse or absent, large glandular cells (GC) with many internal vacuoles open through ducts and cuticle channels (CuC).

We can confirm Jordan’s observations of hypodermal gland cells (Class 1, epithelial gland cells without duct cell) that are spread over the entire abdomen, but are more conspicuous on the dorsal than on the ventral side. They are particularly conspicuous in the tergites VII, VIII and IX (Fig 6). In addition, especially at the lateral regions of these tergites, one finds small gland cells of class 3 (Fig 6C). In contrast to Jordan [6], we cannot recognize a significant difference in the cuticular glandular endowment of *Lomechusoides* and *Lomechusa*, albeit the trichome area in the abdominal segments III, IV, and V of *Lomechusoides* is more richly endowed with trichome setae which reach from the tergal lateral edges to almost the tergal center line (see Fig 2).

**Fig 6:** Longitudinal sections through the abdominal tip of *Lomechusoides strumosus*. (a) Overview of the abdominal tip. Part of the post-pleural gland (PplG) is visible. (b) Close-up of tergites VIII and IX, showing the well-developed glandular epithelium (GE) in both segments. (c) Close-up view of tergite IX showing the cylindrical glandular cells in glandular epithelium (GE). (d) Glandular cells (GC) with ducts at the edges of tergite VIII.

In the 7^th^ and 8^th^ abdominal segments of both genera exist paired clusters of glandular cells (class 3) the ducts of which open as bundles in the pleural area through the intersegmental membrane between abdominal segment VIII and IX (Figs 7, 8 and 9). We think that these glands are identical to those Pasteels [20] calls post-pleural glands. In cross sections we could clearly determine the duct openings through the pleural intersegmental membrane. As Pasteels already noted, Jordan [6] did not recognize these glands. Pasteels also mentions”very thick” glandular cells with ducts deeply submerged inside the body along the major tracheal tracts. He suggests that they open at the lateral corners of the third and fourth tergites. It is not clear to us whether his findings refer to the glandular cell bundles that open through the cuticle near the tracheal strand that leads to the spiracle. They are particularly large in the third, fourth and fifth tergites, but they are also present, albeit much smaller, in other abdominal segments (see Figs 3 and 4C).

**Fig 7:** Post-pleural gland in *Lomechusoides strumosus*. (above) Glandular cells (GC) and ducts that open in densely packed pores (GDO) in the pleural intersegmental membrane. (below) Large glandular cells (GC) with duct cells (DC).

**Fig 8:** Post-pleural gland and other glandular structures in the abdominal tip of *Lomechusa pubicollis*. (a) Post-pleural gland with glandular cells (GC) and duct cells (GD) opening through the pleural intersegmental membrane between the abdominal segment VIII and IX. (b, c). large glandular cells (GC) in the posterior part of the abdomen with large intra-cellular reservoirs (GR).

**Fig 9:** Scanning electron microscopic images of the abdomen of *Lomechusoides strumosus*. PLG: opening of the post-pleural gland. DTG: opening of the defense tergal gland.

We assume, however, Pasteels [20] might refer to the truly “thick” glandular cells with ducts and intracellular reservoirs we find in the posterior abdominal part, both in *Lomechusoides* and *Lomechusa*. They are particularly obvious in species of the latter genus, including *Lomechusa pubicollis* and *L*. *emarginata* (Fig 8B and 8C). We were unable to determine exactly where they open, but it must be in the posterior part of the abdomen and they might even be part of the post-pleural gland complex.

The most obvious abdominal gland structure in *Lomechusoides* as well as *Lomechusa* is the composite tergal gland. It was first discovered and described by Jordan [6], later confirmed by Pasteels [20] and Hölldobler [11]. The gland consists of two glandular systems. 1) Paired clusters of large secretory cells of class 3 with long ducts that open through an extended cuticle ridge on the anterior edge of the 7^th^ abdominal tergite, leading into paired pouches that are formed by invagination of the intersegmental membrane between the 6^th^ and 7^th^ tergites. 2) Part of the membrane of the reservoir pouches is a massively developed glandular epithelium, consisting of glandular palisade cells (Fig 10). Jordan identified this correctly as a defensive gland. Blum et al. [23] found the tergal gland secretion of *Lomechusoides strumosus* to contain benzoquinone, methyl-benzoquinone, ethyl-benzoquinone and n-tridecane, the later substance accounting for more than 80% of the volatiles detected in the secretion. The schematic drawing in Fig 11 gives an overview of the exocrine glands found in the abdomen of *Lomechusoides*.

**Fig 10:** Longitudinal section through the defense tergal gland of *Lomechusoides strumosus*. (top) The complex gland structure consists of the glandular cells (GC) with duct cells (D) that open through the cuticle of the 7^th^ abdominal tergite into a reservoir (R). Part of the reservoir membrane is a glandular epithelium (GE). (bottom) Close-up of the glandular epithelium (GE) showing the large cylindrical glandular cells.

**Fig 11:** Schematic illustration of the major exocrine glands in the abdomen of *Lomechusoides strumosus*. The green area of abdominal segments II to V is the adoption gland complex (AG). Between abdominal segments VI and VII is the defense tergal gland or repellent gland, the reservoir (Re) of which opens between these two segments. The repellent secretion is a mixture of the secretions of the glandular epithelium (RGE) and the glandular cells (RGC). PlG indicates the location of the post-pleural gland. HG: hindgut; R: rectum. The blue area indicates the appeasement gland complex.

*Lomechusoides* beetles are also richly endowed with epithelial glands on the edges of the prothoracic shield and head. We found glandular cells in the frontal head area and ventral near the mandibles, inside the mandibles, the labrum and labium (Fig 12) and as a glandular epithelium in the basal segments of the antennae (Fig 13).

**Fig 12:** Longitudinal sections through the head of *Lomechusoides strumosus*. (a) Overview of part of the head. Br: brain; M: muscle; GC: glandular cells near the base of the mandibles. (b) Close-up of these gland cells that open through the cuticle channels (CuC). (c) Longitudinal section through the mouth parts. Lbr: labrum; M: mandible, with an epithelium consisting of sensory and glandular cells (GC/SC) in the posterior. Ga: galea. (d) Glandular cells (GC) in the labium (Lab).

**Fig 13:** Glandular epithelium (GE) in antennal segments of *Lomechusoides strumosus*.

The glandular ducts of these hypodermal cells in the head and abdomen open through pore plates or singular pores (Fig 14). All such glandular structures are also present in the species *L*. *pubicollis* and *L*. *emarginata*. An astonishing difference between both genera is the generous endowment with glandular cells in the legs of *Lomechusoides*. In fact, the femur of the three pairs of legs of *Lomechusoides* are equipped with trichomes associated with densely packed glandular cells (Figs 15, 16 and 17). Glandular cells are also found in the tibia. In *Lomechusa* some glandular cells can also be found in the legs, however, these are much less conspicuous and leg trichomes are absent.

**Fig 14:** Scanning electron microscopic images of the cuticle glandular pores of *Lomechusoides strumosus*. (a) Labrum with densely spaced pore plates (GPpl). (b) Close-up of cuticle of the 8^th^ abdominal tergite. Many of the pore plates and pores (GP) are less than 10 μm apart. (c) Close-up of a glandular pore plate. Its diameter is less than 2 μm.

**Fig 15:** **Scanning electron microscopic images of the side view of *Lomechusoides strumosus* (a) and *Lomechusa pubicollis* (b)**. Close-up of the femur (Fe) of *L*. *strumosus* (c); the trichome setae are clearly visible. (d) Close-up of the femur of *L*. *pubicollis*. Trichome setae are absent.

**Fig 16:** Trichome glands in the femur of *Lomechusoides strumosus*. (above) Scanning electron microscopic image of the ventral side of the femur. Box indicates the location of the histological preparation shown in bottom panel. (below) Glandular cells (GC) inside the femur.

**Fig 17:** Longitudinal sections through the leg of *Lomechusoides strumosus*. (a) and (c) Longitudinal sections through the femur showing the densely packed glandular cells (GC) with the cuticle channels (CuC). (b) and (d) Longitudinal sections through tibia proximate to the femur, showing the dense layer of gland cells with ducts through the cuticle.

Finally, we briefly describe the gut system, because our behavioral studies indicate that especially the hindgut might be involved in the beetles’ interactions with the host ants. Inside the crop, there exist relatively densely packed, long sclerotized bristles that point towards the proventriculus (Fig 18, above). The proventriculus is a short muscular structure that regulates the flow from crop into the midgut. The midgut is endowed with many caecal diverticula, and the hindgut epithelium is thick, the cells of which have large nuclei and appear to be secretory cells (Fig 19).

**Fig 18:** Longitudinal section through part of the alimentary tract of *Lomechusoides strumosus*. (above) Crop (Cr) and proventriculus (PrV). The crop is lined with layers of longitudinal and transversal muscles, and in the lumen the sclerotized spines are visible. (below) The transition from crop via proventriculus to midgut (MG). The midgut is endowed with many diverticula (DiV) along its entire length.

**Fig 19:** Sections through the hindgut of *Lomechusoides strumosus*. (a) Longitudinal section through the hindgut (HG) and rectum (R). (b) and (c) Transversal sections showing the large gland cell nuclei (GCNu) in the hindgut epithelial cells (HGE). (M) Muscle tissue surrounding hindgut layer. (d) Transversal section of hindgut showing the microvilli structure (MiVi) of the hindgut cells.

### Adoption behavior

Wasmann (summarized in [8, 9]) and also Jordan [6] provide many descriptions of the behavioral interactions between the *Lomechusoides* beetles and their host ants, but they did not describe the adoption process of the beetle by its host ants. This was studied in detail in *Lomechusa pubicollis* by Hölldobler [11, 24] but until now, little has been known about adoption in *Lomechusoides*.

When we placed a beetle collected from a field colony in the arena of a laboratory colony we noticed that the beetle, when contacted by an ant, positioned its legs outward so that the relatively large femurs reached out in an almost horizontal position. Usually the ants licked the legs, in particular the femurs. The beetle bends backward or sideward with head and thorax, apparently in attempt to contact the ant with its antennae (Fig 20). It often rolls up its abdomen and points the tip of it toward the ant. Our more detailed observations of the first 15-minute encounter-phase showed that at the beginning the ants often exhibited a somewhat aggressive behavior, and previous authors (i.e. Wasmann, Jordan) interpreted the curling up of the abdomen by the beetles as a behavior connected with the discharge of the repellent secretion from the defense tergal gland. However, during our observations, we hardly ever noticed the beetle discharging the repellent secretion (which can be easily smelled) when encountering potential host ants. Instead, the beetle exhibited slight turns and waggle movements when an ant approached it sideways. In this way the ants first contacted the leg of the beetle, and simultaneously the beetle bent backwards and sideways seeking contact with the ants with its antennal tips, the last segments of which are packed with chemo-sensilla.

**Fig 20:** Adoption process in *Lomechusoides strumosus*. At first encounter the ants often lick the distal part of the beetle’s extended femur (above) or the proximate part of the beetle’s tibia (below).

We often observed that the ants that initially exhibited some aggressive behavior started to lick the abdominal tip of the beetle whilst the beetle continued to reach backwards (Fig 21). Frequently, but not regularly, a white, opaque, droplet appeared at the abdominal tip, most likely the opening of the rectum, but in some cases, we also noticed translucent, whitish secretions appearing at the lateral spot where the post-pleural gland opens (Fig 22).

**Fig 21:** Adoption process in *Lomechusoides strumosus*. The abdominal tip is the most frequently encountered body part of the beetles which the prospective host ants inspect and lick. During this process the beetle attempts to touch the ant with its antennal tip (b, c, d). Finally, the beetle unrolls its abdomen (e, f) while the ants continue to lick the abdominal tip.

**Fig 22:** Appeasement substance. (above) Often the beetle exudes an opaque, white droplet from its abdominal top, which is taken up by the ant. Presumably it originates from the hindgut/rectum. (below) Occasionally a whitish, clear secretion appears at the lateral sides of the abdomen where the post-pleural gland opens. This secretion is also licked by the ants.

The results show that in the initial encounter phase, the ants contact the posterior of the beetle’s abdomen most frequently, followed by the leg (Fig 23). Only after this initial phase, which can last 5–20 minutes, do the beetles allow the ants to have full access to the tufts at their abdominal margin (Fig 24). Finally, an ant grabs the beetle at the trichome tufts and lifts it upward. The beetle assumes a pupal position with the appendages folded tightly to the body and the beetle is carried into the nest, where it finally “takes residence” in the brood chamber (Fig 25). Occasionally we observed beetles approaching the nest entrance and entering the nest on their own. Inside they may subsequently be picked up by a nest worker and carried into the brood chamber.

**Fig 23:** Parts of the beetle body contacted prior to adoption. We recorded the number of times ants contacted various body regions of newly introduced beetles (n = 10). The beetle’s abdominal tip and legs received the highest and second highest proportion of contact, respectively (bars are means with standard error).

**Fig 24:** Adoption process in *Lomechusoides strumosus*. After aggressive behavior of the ants has waned due to the appeasement behavior (a), the beetle allows the ant to access the adoption glands (the trichome area at the margins of the first abdominal segments; b, c, d).

**Fig 25:** Adoption process in *Lomechusoides strumosus*. In the last phase of the adoption process the ant grasps the beetle on the trichome hairs and lifts it up. The beetle assumes a pupal position and is carried into the nest.

### Trophallactic interactions

The participation of *Lomechusoides* beetles in the food flow inside the host ant colony has been known since Wasmann’s extensive studies. One can frequently observe mouth-to-mouth contact between the beetles and ants, and, by marking the food provided to the ants with a dye and subsequent dissections, Wasmann demonstrated that food was transferred from ant to beetle.

The application of the radioactive tracer technique allowed us to obtain more quantitative data. Observations indicated that frequency and duration of trophallactic contacts between ants and beetles differed between groups where beetles were housed with familiar “nestmate” ants or with unfamiliar ants from a foreign host colony. In our test groups, the ants consumed an equivalent amount of labeled food before the beetles were introduced (t_30_ = -1.79, P = 0.48, familiar *F*. *sanguinea* mean of within group averages: 746 Imp/100sec (SD 226), unfamiliar *F*. *sanguinea* mean of within group averages: 880 Imp/100sec (SD 183)). After 24-hrs spent together, there was no significant difference between familiar beetles and ants, indicating that familiar beetles obtained a large amount of food from the host ants, equivalent to that shared between the host workers themselves (dependent t-test comparing familiar ants and familiar beetles, not significant: t_36_ = 0.70, P = 0.49). In the groups with unfamiliar ants, the beetles obtained some food, but had significantly less than their unfamiliar hosts after 24-hrs. Unfamiliar beetles showed only 10.4% of the average amount of food each of the host ants carried (Independent t-test comparing unfamiliar ants and unfamiliar beetles, significantly different: t_24_ = 14.38, P < 0.0000) (Fig 26). Most likely, the beetles acquire the host colony’s specific nest odor by the frequent close contact with the ants during the adoption interactions.

**Fig 26:** Ants preferentially shared food with familiar beetles. Beetles fed with labeled honey water were placed with familiar or unfamiliar beetles. Beetles from both groups successfully obtained food from their host ants, but familiar beetles obtained significantly more food than unfamiliar beetles (bars are means with standard errors).

In tests to determine whether food is transferred from fed beetles to ant hosts, we found that beetle impulse counts remained significantly higher than those of their ant hosts across the 48-hr sampling period (LMM, t = -30.14, P < 0.00001, Fig 27). However, there was a significant interaction between species identity and the final sampling event, due to a slight increase in impulse counts for some ants after 48 hours (LMM, t = 2.74, P = 0.0012). While there is a clear transfer of liquid food from ants to beetles, this experiment demonstrates that beetles are unlikely to transfer food back to ants. After 48 hours, just 4% of the average food inside the beetles was shared with the ants. Instead of engaging in trophallaxis, ants likely consumed small amounts of beetle feces or secretions. In fact, the following results strongly suggest that the ants may have consumed some of the white secretion which appears to be ejected by the beetles from the rectum.

**Fig 27:** Beetles did not share food directly with ants, over time. Over 48-hrs, beetles that fed on labeled food emitted significantly higher impulse counts than the ants they were housed with (LMM, P < 0.00001). Beetles lost a small proportion of their signal, while ants obtained a significant (but low-level) signal between the first final sampling periods (LMM, P < 0.0026), possibly from consuming beetle feces or excretions. Each trial (n = 4) is represented by a different color. Beetle impulse counts are represented by open circles, and associated ants with closed circles.

Beetles that previously received labeled honey-water emitted an average of 1,090 impulses/min (SD 150). Abdominal tip secretions emitted significantly more impulses/min than control cotton buds alone (control mean = 20.14, secretion mean = 51.29, dependent t-test, t_6_ = -6.34, p = 0.00072). The amount of radioactive material collected from abdominal tip secretions was not significantly different from the amount obtained by some ants after they spent 48 hours with beetles that had been fed with labeled honey-water (independent t-test, t_9_ = -2.02, p = 0.080).

Wasmann and others observed the food exchange behavior between adult *Lomechusoides* beetles and host ants, and noted that in contrast to *Lomechusa* (*Atemeles*), *Lomechusoides* does not use the forelegs to stimulate the host ants’ regurgitation (see also [11, 24]). In *Lomechusoides* the ants’ behavior often resembles that which the ants exhibit when feeding ant larvae or the beetle larvae [10]. The antennae are often pointed towards the head of the beetles and the mandibles are closed (Fig 28).

**Fig 28:** Trophallaxis between *Lomechusoides strumosus* and host ant *Formica sanguinea*. Often the ant approaches the beetle and licks its head (a). The beetle seeks contact with the ant’s labium (b, c). This usually leads to regurgitation of food by the ant. During the trophallactic act shown in (d), the ant’s mandibles are closed, but the labium is extended. This somewhat resembles the feeding behavior which ants exhibit during larval feeding.

However, we have also observed the typical “donor-behavior” in ants when feeding a beetle, identical to that which they exhibit in trophallaxis with ant nestmates: widely gaping mandibles, labium extended and antennae folded backwards (Fig 29, above). Occasionally one can observe two beetles standing head to head, as if conducting trophallaxis (Fig 29, below). However, our tracer experiments did not reveal any indication that food exchange occurred between *Lomechusoides* beetles.

**Fig 29:** Trophallaxis interactions in *Lomechusoides strumosus*. The host ant *Formica sanguinea* regurgitates food to the beetle (above). The ant’s mandibles are opened, the labium is extended. This resembles the feeding behavior among adult ants. (below) Occasionally two beetles have mouth to mouth contact, however we could not find evidence that they exchange food.

In this context it is worthwhile to mention that the mouthparts of *Lomechusoides* and *Lomechusa* show a number of features that may be important tools to stimulate ant regurgitation. In his revision of the genus *Lomechusa*, Hlaváč recognizes that in this genus, the galea of the maxilla is larger than the lacinia. We confirm that this is also the case in *Lomechusoides*. In addition, the galea is equipped with densely packed, long bristles and also the lacinia has many bristles, albeit not as long and bent as those if the galea (Fig 30). Furthermore, both *Lomechusoides* and *Lomechusa* have an unusually large prostheca of the mandible, which is endowed with a brush-like, fringed selvedge composed of several cuticle layers (Fig 31). It is conceivable that these mouthpart structures support the beetles’ stimulation of the ant’s labium that releases regurgitation in the ant. The related aleocharine *Pella* sp. which hunts ants or feeds on corpses along the trunk routes and kitchen middens of the ant species *Lasius fulginosus* [25], has a much smaller prostheca (Fig 31) and the maxillar mouthparts are not as richly endowed with bristles as those of *Lomechusoides*. In his studies of the mouth parts of *Lomechusoides* and *Lomechusa* beetles. Wasmann [26] paid little attention to the maxillae, but noticed that the labium is shortened and broader particularly in *Lomechusoides*; it is fused with the paraglossae, and the number of segments of the labial palps are reduced. In this way, the labium looks more like a spoon than a tongue, and Wasmann considered this a special adaptation of the beetles being fed by the host ants.

**Fig 30:** Scanning electron microscopic images of the mouth parts of *Lomechusoides strumosus*. (left) Close-up of ventral view of galea (Ga) and lacinia (La) of the maxillae. (right) Dorsal view maxillary palps (MP), galea (Ga), and mandibles (Ma).

**Fig 31:** Scanning electron microscopic images of the mandibles of three aleocharine beetle species. *Lomechusoides strumosus* (a) and *Lomechusa pubicollis* (b) both have a large protheca (PT) in contrast to *Pella sp*. (c) where the protheca is much smaller.

## Concluding results and discussion

Many species of insects and other arthropods live with ants and have developed a thriving parasitic relationship with them. The staphylinid beetle species *Lomechusoides strumosus* is arguably one of the most thoroughly studied examples, due to the careful observations of Erich Wasmann during a period of three decades (overviews of Wasmann’s publications [8, 9]). Wasmann discovered many phenomena regarding the natural history of *L*. *strumosus*, he also attempted to understand the evolution of this intricate parasitic-symbiotic relationship of the myrmecophile and its host ants *Formica sanguinea*. He proposed that the ants evolved a special symphilic instinct, an aberration of the brood care instinct. He also argued that the host ants are actively selecting the most desirable beetle individuals for breeding the myrmecophiles, because the ants became “addicted” to the glandular secretions exuding from the “trichome glands.” He termed this specific selection behavior “amical selection.” Although Wasmann’s hypothesis was attacked by several contemporary entomologists [6, 27, 28], Wasmann responded listing many behavioral facts he assembled, which he thought solidly supported his theory. Finally, in 1948 K. Hölldobler [29] published a detailed analysis of the facts and theoretical arguments Wasmann listed, concluding that although the facts are not in question, Wasmann’s evolutionary interpretation lacked a logical foundation. Nevertheless, even he proposed that the ant hosts might eventually develop a kind of “addiction” for the trichome exudate, and therefore tolerate the beetles, despite the fact that they can become detrimental to the colony. Indeed, Wasmann found a strong correlation of aberrant worker morphology (so-called pseudogynes) and striking decline of the production of alate reproductives in colonies that house *L*. *strumosus*. Although the exact physiological cause of the aberrant development of workers and decline of production of sexuals is not known, given that the beetles are diverting food from the colony, it is likely this phenomenon is caused by starvation of the larvae. It should also be pointed out that the correlation between the occurrence of *Lomechusoides* larvae and pseudogynes in *Formica sanguinea* colonies could not be confirmed by Donisthorpe [30]. However, Donithorpe himself states that his data base is by far not as extensive as that of Wasmann. In summary K. Hölldobler recognized that the myrmecophiles exploit stimuli the ants employ in intraspecific interactions within the colony, and called the myrmecophilous beetles “psychoparasites”.

Based on our experimental investigations of *Lomechusa* (formerly *Atemeles*) *pubicollis* [10, 11, 24] and the present work on *Lomechusoides* (formerly *Lomechusa*) *strumosus*, we conclude that these myrmecophiles have broken the ants’ communication code. They most likely mimic the ants’ brood tending pheromones, and parasitize the innate releasing mechanism of the hosts’ brood tending behavior. In *Lomechusoides*, not only are the beetle larvae treated like ant larvae [10], but also the adults. As our current work demonstrates in detail that the adult beetles, once accepted by the ants, are carried by the ants into the brood chambers, where the beetles prey on the ant brood and are fed by the ants. We do not know whether the food quality is different when beetles are fed in “larva mode” or adult trophallactic mode, although we registered the transfer of radioactively labeled food in both situations. It is possible that in the “larval mode” contents from the labial gland are also fed to the beetle. In *Lomechusa pubicolis*, we previously demonstrated that the larvae as well as the adult beetles obtain more food from the workers than both ant brood and worker nestmates do. This is also the case in *Lomechusoides*. The larvae receive more food from their host ant nurse worker [10] than the host larvae, and the results reported in the current paper indicate that this might also be true for adult beetles.

All of this suggests that the social parasitism of *L*. *strumosus* is based on the supernormal imitation of the brood tending releaser, a chemical signal that the adult beetles exude from the “trichome glands.” In both *Lomechusa pubicollis* and *Lomechusoides strumosus*, these glands play a critical role in the adoption process of the beetle. Therefore, we call these structures “adoption glands” [11, 24]. During the adoption process, glands in the abdominal tip, which closely resemble those of *Lomechusa pubicollis* beetles and which Hölldobler [11, 24] has called appeasement glands, serve as gentle defense tools. We think that the post-pleural gland (first correctly identified by Pasteels [20]), the hypodermal gland epithelia in the VIII^th^ and IX^th^ tergites and sternites are part of the appeasement gland complex, and we suggest that the glandular hindgut, with is contents, also contributes to the appeasement process. Initially, aggressive ants that contact the posterior part of the beetle’s abdomen with their mouthparts lick the tip, terminal tergites, and sternites and imbibe whitish droplets that often appear at the opening of the rectum during the ant-beetle interactions. Previous authors [8] interpreted the upward raising of the abdominal tip as an indication that the beetles discharge a repellent substance from the defensive tergal gland. We never observed this defense response during encounters with the host ants, but noticed it when beetles came in contact with other ant species. During interactions with host ants the bending upwards of the beetles’ abdomen is in most instances a presentation of the appeasement gland complex.

The trichomes and glands of the legs (especially the femur) of *Lomechusoides strumosus* beetles seem to be unique to the genus. They are absent in *Lomechusa* and most likely also in *Xenodusa*, the third genus of the subtribe Lomechusina. This latter genus is the only one that occurs in the Nearctic region [12]. Our observations indicate that these structures, employed during first encounters with ants, serve as a first “gentle” barrier for ants seeking access to the abdominal trichome glands (adoption-glands). Indeed, once the ants reach the adoption glands of beetles outside the nest, they grab the beetle on the trichome tufts and carry it into the nest. This behavior appears to be identical to that observed in *Lomechusa pubicollis* by Hölldobler [11, 24].

The adoption behavior is a key factor in the parasitic relationship of *Lomechusoides* to its hosts, because during the beetle’s life trajectory, it has to seek acceptance by different host ant colonies. As Wasmann pointed out in several of his studies (see [8, 9]), the beetle migrates several times from one host colony to another as an adult. After reaching sexual maturity in the *Formica sanguinea* nest, in which the larvae have been raised, the beetles leave the host nest and emigrate to another one where they meet conspecifics that were raised in different *F*. *sanguinea* nests. As Wasmann observed, one male (recognizable by the hair tufts on the third and fourth antennal segments, Fig 32) can mate with several females, and a female often mates with several males (Fig 33). She stores the sperm in a large, sclerotized spermatheca (Fig 34), typical of many aleocharine staphylinids [31]. After mating, some beetles migrate again to yet another *F*. *sanguinea* nest, where their larvae will be raised. In each case, the beetles have to ease in their entry to a foreign colony, which is greatly facilitated by the complex adoption behavior. Wasmann assumed that the beetles might be ovoviviparous, because he never found *Lomechusoides* eggs in the host ants’ nest, but sometimes discovered first-instar beetle larvae on the egg piles of the ants. Our histological work does not indicate any sign of ovovivipary. Perhaps the beetle eggs are physically indistinguishable from the ant eggs, and therefore impossible to discover in the egg pile of the ants.

**Fig 32:** Scanning electron microscopic images of the head and antennae of male *Lomechusoides strumosus*. (a,b,c,d,) Different views and magnifications of the typical hair tufts (AT) the beetle males display on their third and fourth antennal segments.

**Fig 33:** Mating in *Lomechusoides strumosus*.

**Fig 34:** Spermatheca of *Lomechusoides strumosus*. (left) The sclerotized spermatheca (SpT) and spermathecal gland (SpTG). (right) Close-up of the spermatheca gland (SpTG) showing the densely packed duct cells (SpTGD).

June and July are the larval period of *Lomechusoides* and the pupal period stretches from end of July to beginning September. This includes several reproductive bouts of the year’s beetle generation. The dirt covered pupal cells are hidden in the soil of the nest; when discovered by the ants, they are usually thrown out of the nest. The first young beetles were found in August and beginning September. Our observations from our collecting sites in Franconia do not exactly match Wasmann’s [8] quantitative field data collected in the Netherlands, but they are close. In these freshly eclosed *Lomechusoides* beetles’ spermatogenesis and oogenesis is still in progress. The young beetles overwinter in the host ant nest, and some of them may actually leave the nest where they were raised and migrate to another one for overwintering [8]. We did not find evidence for such migrations in the fall.

Like in *Lomechusoides* the life trajectories of *Lomechusa* beetles are also characterized by migrations between host colonies, but unlike *Lomechusoides*, *Lomechusa* changes not only host colonies, but also host species [8, 9, 11, 24]. After the *Lomechusa* larvae have pupated and hatched in the Formica nest, the adult beetles migrate in the fall to nests of the genus *Myrmica*, and in spring, they return to the *Formica* colonies. Hölldobler [11] suggested that the life cycles of *Lomechusa* beetles is adapted to that of *Formica* and *Myrmica* ants, so that the beetles can take maximum advantage of the social life of both host species. It appears that *Lomechusa*, like *Lomechusoides*, evolved myrmecophilous relations with *Formica* first and subsequently adapted to the winter host *Myrmica*, because *Myrmica*, in contrast to *Formica*, overwinters with brood, which secures a rich food source for the beetles needed for the completion of its sexual maturity.

## References

[1] WilsonEO. The Insect Societies: Harvard University Press; 1971.

[2] HölldoblerB. Verhaltensphysiologische Adaptationen an ökologischen Nischen in Ameisennestern. Verhandlungsbericht der Deutsch Zool Ges. 1972;65:137–43

[3] HölldoblerB, WilsonEO. The Ants Cambridge, MA: Harvard University Press; 1990.

[4] ParkerJ. Myrmecophily in beetles (Coleoptera): Evolutionary patterns and biological mechanisms. Myrmecological News. 2016;22:65–108.

[5] HölldoblerB, KwapichCL. *Amphotis marginata* (Coleoptera: Nitidulidae) a highwayman of the ant *Lasius fuliginosus*. PLOS ONE. 2017;12(8). 10.1371/journal.pone.0180847 28783744PMC5546582

[6] JordanKHC. Zur Morphologie und Biologie der myrmecophilen Gattungen *Lomechusa* und *Atemeles* und einiger verwandter Formen. Zeitschrift Vergleichende Physiologie. 1913;107:346–86.

[7] WasmannE. Zur näheren Kenntnis des echten Gastverhältnisses (Symphilie) bei den Ameisen- und Termitengästen. Biolisches Zentralblatt. 1903;23:63–27; 195–207; 32–48; 61–76; 98–310.

[8] WasmannE. Neue Beiträge zur Biologie von *Lomechusa* und *Atemeles*, mit kritischen Bemerkungen über das echte gastverhältnis. Zeitschrift fur Wissenschaftliche Zoologie. 1915;114:233–402.

[9] WasmannE. Die Gastpflege der Ameisen Berlin: Gebrüder Borntraeger; 1920.

[10] HölldoblerB. Zur Physiologie der Gast-Wirt-Beziehung (Myrmecophilie bei Ameisen. I. Das Gastverhältnis der *Atemeles*-und *Lomechusa*-Larven (Col. Staphylinidae) zu *Formica* (Hym. Formicidae). Zeitschrift Vergleichende Physiologie. 1967;56:1–21.

[11] HölldoblerB. Zur Physiologie der Gast-Wirt-Beziehung (Myrmecophilie bei Ameisen. II. Das Gastverhältnis der imaginalen *Atemeles pubicollis* Bris. (Coleoptera: Staphylinidae) zu *Myrmica* and *Formica* (Hymenoptera: Formicidae). Zeitschrift Vergleichende Physiologie. 1970;66:215–50.

[12] HlaváčP. Revision of the myrmecophilous genus *Lomechusa* (Coleoptera: Staphylinidae: Aleocharinae). Sociobiology. 2005;46:203–50.

[13] SawadaK. New myrmecophilous Coleoptera in Nepal and Japan (Histeridae & Staphylinidae). Contributions from the Biological Laboratory, Kyoto University 1994;28:357–65.

[14] SchilowWF. Taxonomische Bemerkungen űber die Kurzflűgler der Gattung *Atemeles* aus der UdSSR (Coleoptera, Staphylinidae, Aleocharinae). Reichenbachia 1977;16:323–6.

[15] SchilowWF. Die *Lomechusa*-Arten der Sowjetunion und angrenzender gebiete (Coleoptera: Staphylinidae, Aleocharinae). Reichenbachia. 1981;19:213–23

[16] SchilowWF. Eine neue Art myrmecophiler Käfer aus der Tadshikischen SSR (Coleoptera, Staphylinidae, Aleocharinae). Deutsche Entomologische Zeitschrift, 1997;24:371–2.

[17] GößwaldK, KloftW. Neuere untersuchungen über die sozialen wechselbeziehungen im ameisenvolk, durchgeführt mit Radioisotopen. Zoologische Beiträge NF. 1960;(5):519–56.

[18] Romeis B. Mikroskopische Technik. Munich1948.

[19] RathmayerW. Paralysis Caused by the Digger Wasp *Philanthus*. Nature. 1962;196:1148 10.1038/1961148a0

[20] PasteelsJM. Le systeme glandulaire tegumentaire des Aleocharinae (Coleoptera, Staphylinidae) et son evolution chez les especes termitophiles du genre *Termitella*. Archives de Biologie (Liege). 1968;79:381–469.

[21] NoirotC, QuennedeyA. Fine structure of insect epidermal glands. Annual Review of Entomology. 1974;19(1):61–80. 10.1146/annurev.en.19.010174.000425

[22] BillenJ. Exocrine Glands and Their Key Function in the Communication System of Social Insects. Formosan Entomology. 2011;31:75–84.

[23] BlumMS, CreweRM, PasteelsJM. Defensive secretion of *Lomechusa strumosa*, a myrmecophilous Beetle. Annals of the Entomological Society of America. 1971;64(4):975–6. 10.1093/aesa/64.4.975

[24] HölldoblerB. Communication between ants and their guests. Scientific American. 1971:86–93.5538697

[25] HölldoblerB, MöglichM, MaschwitzU. Myrmecophilic Relationship of *Pella* (Coleoptera: Staphylinidae) to *Lasius fuliginosus* (Hymenoptera: Formicidae). Psyche. 1981;88(3–4):347–74. 10.1155/1981/75317

[26] WasmannE. Zur Biologie und morphologie der *Lomechusa*-gruppe. Zoologischer Anzeiger. 1897;20:463–71.

[27] EscherichK. Zur Anatomie und Biologie von *Paussus turcicus* Friv., zugleich ein. Beitrag zur Kenntniss der Myrmecophilie. Zoologische Jahrbücher Abteilung für Sys- tematik, Geographie und Biologie der Tiere) 1898;12:27–70.

[28] WheelerWM. Ants New York: Columbia University Press; 1910 696 p.

[29] HölldoblerK. Über ein parasitologisches Problem: Die Gastpflege der Ameisen und die Symphilieinstinkte. Zeitschrift für Parasitenkunde 1948;14:3–26.

[30] DonisthorpeHSJK. The Guests of British Ants Their Habits and Life-histories. London: George Routledge And Sons, Limited 1927 244 p.

[31] GackC, PeschkeK. Spermathecal morphology, sperm transfer and a novel mechanism of sperm displacement in the rove beetle, *Aleochara curtula* (Coleoptera, Staphylinidae). Zoomorphology. 1994;114(4):227–37. 10.1007/bf00416861

